The article "Psychedelics and Psychotherapy: Cognitive-Behavioral Approaches as Default" was published in 2022. Journal: Front Psychol.

# Psychedelics and Psychotherapy: Cognitive-Behavioral Approaches as Default

**DOI:** 10.3389/fpsyg.2022.873279

**Published:** 2022-05-23

**Authors:** David B. Yaden, Dylan Earp, Marianna Graziosi, Dara Friedman-Wheeler, Jason B. Luoma, Matthew W. Johnson

**Affiliations:** ^1^Department of Psychiatry and Behavioral Sciences, Johns Hopkins University School of Medicine, Baltimore, MD, United States; ^2^Department of Psychology, University of California, Berkeley, Berkeley, CA, United States; ^3^Department of Clinical Psychology, Hofstra University, Hempstead, NY, United States; ^4^Portland Psychotherapy Clinic, Research, and Training Center, Portland, OR, United States

**Keywords:** psychedelics, psilocybin, LSD, psychedelic assisted therapy, cognitive behavioral therapy (CBT), dialectical behavior therapy (DBT), acceptance and commitment therapy (ACT), psychedelic assisted psychotherapy

## Abstract

The acute subjective effects of psychedelics are responsive to users’ expectations and surroundings (i.e., “set and setting”). Accordingly, a great deal of thought has gone into designing the psychosocial context of psychedelic administration in clinical settings. But what theoretical paradigms inform these considerations about set and setting? Here, we describe several historical, sociological influences on current psychedelic administration in mainstream European and American clinical research settings, including: indigenous practices, new age spirituality from the 1960s, psychodynamic/psychoanalytic approaches, and cognitive-behavioral approaches. We consider each of these paradigms and determine that cognitive-behavioral therapies, including newer branches such as acceptance and commitment therapy (ACT), have the strongest rationale for psychedelic-assisted psychotherapy going forward. Our primary reasons for advocating for cognitive-behavioral approaches include, (1) they avoid issues of cultural insensitivity, (2) they make minimal speculative assumptions about the nature of the mind and reality, (3) they have the largest base of empirical support for their safety and effectiveness outside of psychedelic therapy. We then propose several concepts from cognitive-behavioral therapies such as CBT, DBT, and ACT that can usefully inform the preparation, session, and integration phases of psychedelic psychotherapy. Overall, while there are many sources from which psychedelic psychotherapy could draw, we argue that current gold-standard, evidence-based psychotherapeutic paradigms provide the best starting point in terms of safety and efficacy.

## Introduction

Classic psychedelics, such as 5-HT2a partial agonist psilocybin, are being tested for their potential therapeutic effects. Psilocybin is well-tolerated in clinical settings in which precautions have been taken to screen out participants who might have medical or psychological contraindications and where clinicians are available to provide support (Johnson et al., 2008). In general, the risks of toxicity and addiction are comparatively low with psilocybin compared to other recreational psychoactive substances (Johnson et al., 2008; Nichols, 2016), though there are risks to psychedelic use in general which are increased in recreational settings (Carbonaro et al., 2016). Clinical trials have demonstrated the therapeutic potential of psilocybin on both mood (Carhart-Harris et al., 2016, 2021; Griffiths et al., 2016; Ross et al., 2016; Davis et al., 2021) and substance use disorders (Johnson et al., 2014; Bogenschutz et al., 2015). Further safety and effectiveness trials are needed (Yaden et al., 2021d), but it is possible that psilocybin (and perhaps other classic psychedelics) will be approved for clinical use in the next few years. While current psychotherapeutic and pharmacological treatments are effective, additional treatment options are needed for those suffering from mood and substance use disorders.

Classic psychedelics present a number of challenges and opportunities in terms of their clinical application. Importantly, the acute subjective effects of classic psychedelics such as psilocybin are highly responsive to one’s expectations and physical/social surroundings (referred to as “set and setting”; Hartogsohn, 2016). This raises the question—-what psychotherapeutic paradigm(s) should most inform the administration of classic psychedelics such as psilocybin?

In this article, we review several historical, sociological influences on the development of contemporary classic psychedelic administration in mainstream healthcare and clinical research settings in European and American cultural contexts. Specifically, we briefly review indigenous practices, new age spirituality, psychodynamic/psychoanalytic approaches, and cognitive-behavioral approaches. After succinctly evaluating each of these and pointing to several issues with each (although extensive analyses of these paradigms goes beyond the scope of the present article), we focus on cognitive-behavioral therapy (CBT) approaches in more detail (also see Walsh and Thiessen, 2018; Luoma et al., 2019) and suggest that these approaches have the most evidence and rationale for serving as a default therapeutic paradigm to combine with psychedelic treatments in contemporary healthcare contexts. While much of what we discuss will apply to other psychoactive substances (e.g., MDMA, ketamine, DMT, etc.), we focus our discussion on classic psychedelics such as LSD and psilocybin. Lastly, we provide a sampling of concepts from CBT approaches, particularly from so-called “third wave” CBT, that we think can usefully inform the preparation, session, and integration phases of psychedelic-assisted psychotherapy.

## Indigenous Practices

Historically, psychedelics appear to have been ingested in a number of regions across a wide range of cultures for hundreds or even thousands of years (Schultes, 1969; Miller, 2019). The available archeological and anthropological evidence suggests that psychedelics have often been used in ritual settings (and they still are, as discussed below), generally accompanied by the invocation of a society’s religious worldviews by a religious leader (e.g., see Miller, 2019). We refer to this approach as “indigenous practices” as this is the term that has been used most by others in contemporary discourse, although we acknowledge that some may object to the use of the term indigenous term in this context. There are a number of contemporary religious traditions, such as the Peyote Church, in which psychedelic substances are ritually ingested. People who engage in these religious practices have a history of being oppressed by colonialists and in more recent eras by prohibition (e.g., see George et al., 2020).

Some have called for more integration of indigenous practices in contemporary, mainstream psychotherapeutic settings using psychedelics (e.g., Winkelman, 2007). The rationale for this view is that some religious practices may have been honed for many decades in order to maximize the beneficial effects of psychedelics. Proponents of this view might suggest that we ignore practices that have been developed over generations at our peril, as such practices could perhaps benefit participants and patients in contemporary healthcare settings.

We agree that such indigenous contexts should be studied, but we see problems with the view that such practices should be incorporated in secular clinical settings. First and foremost, it could be offensive to decontextualize certain kinds of religious practices and transplant them into secular clinical settings. These practices are usually overseen by elders and traditional healers (Portman and Garrett, 2006) and an abundance of literature urges mental health practitioners to partner with these members of indigenous tribes and nations (Dufrene and Coleman, 1992; King, 2008; Gone, 2010; Trimble, 2010). This could be regarded as a case of cultural appropriation, as there is a power differential and potential to profit from adopting such practices in secular healthcare settings. Thus, there are important moral considerations that would seem to largely or entirely prevent drawing from indigenous practices and requisitioning them for use in contemporary healthcare settings. Additionally, *such practices have not been empirically evaluated in clinical settings, so their safety and effectiveness are mostly unknown*, particularly for individuals who do not share in the worldview associated with such practices. Therefore, applying such practices with the bulk of participants likely to receive treatment in mainstream clinical settings could put participants and patients at increased risk.

Of course, if a participant or patient *already* held these beliefs and chose to interpret their personal experience accordingly (see Graziosi et al., 2021), the therapist should accept this as the patient’s worldview and support this participant without disagreeing or suggesting other metaphysical belief systems. As we will reiterate, therapists should not be promoting their own metaphysical belief system to patients (Moreira-Almeida et al., 2016; Johnson, 2020; Koenig et al., 2020; Yaden et al., in press, 2021a). Overall, we believe that treatment should be adapted to the cultural contexts and identities of those seeking treatment but that directly borrowing from indigenous traditions is not an appropriate means to do so for most patients or practitioners.

## New Age Spirituality

Before the current so-called “renaissance” of psychedelic research in the last decade or so, psychedelics were largely associated in the public and even among researchers with the 1960s (e.g., Pollan, 2019). During this period, psychedelics emerged from the laboratory and were adopted by various sub-cultures, including what has been called “new age spirituality” (e.g., Luhrmann, 2012). New age spirituality is a syncretism of various religions, perhaps especially Hinduism and Vedanta, and involves a set of flexibly defined highly personal beliefs. Such beliefs generally (but not necessarily) involve a divinity of some kind and persistence of consciousness after death (Yaden et al., 2021b). While there was a great deal of research conducted on psychedelics in laboratories all over the US during this period of time, the most high-profile research was conducted at Harvard by professors who were later fired or contract not renewed—Timothy Leary and Richard Alpert (Baumeister and Placidi, 1983). These two researchers explicitly mixed new age spiritual ideals into the therapeutic context in the hopes of enhancing the therapeutic effects of psychedelics (Lattin, 2010).

Some have called for more integration of new age spirituality in contemporary psychotherapeutic settings (e.g., Roberts, 2020). The rationale for this view is that beliefs involving a benevolent all-encompassing divinity that one might encounter and/or connect with appears intuitively likely to reduce the chance for a negative experience and could enhance the beneficial effects of psychedelics. There is in fact good evidence that people report experiences of this kind spontaneously (Yaden et al., 2017b; Griffiths et al., 2019; Davis et al., 2020b). However, the extent to which such experiences are the result of the intrinsic effects of psychedelic substances interacting with innate cognitive/perceptual systems or are culturally constructed from available beliefs and expectations is unknown (see Yaden et al., 2017a). To be clear, we see great potential in studying the interaction of psychedelics with beliefs and practices broadly construed as “spiritual.”

However, we see problems with integrating spiritual worldviews into psychedelic psychotherapy in clinical settings. First, there are serious ethical issues with a therapist imposing their own particular worldview (religious, spiritual, atheistic, or otherwise) on a participant or patient (see Johnson, 2020 for a discussion). Psychedelic substances appear to create a suggestable state (Carhart-Harris et al., 2015), which could put participants and patients in a vulnerable position (Johnson, 2020). Additionally, there has been little research on actively encouraging a spiritual framing of psychedelic experiences in therapeutic settings, which means that adopting such a therapeutic frame has unknown risks (see Johnson, 2020). From a secular clinical perspective, we simply have no expertise or knowledge of ground truth regarding metaphysical or religious questions, and the imposition of such content could be considered an epistemological harm (Letheby, 2021). As in the previous section, if a participant or patient holds such beliefs, choosing to engage with them before, during, or after their experience is entirely appropriate and is not the topic under discussion. This does not include the provision of knowledge or expertise but rather taking the patients lead and, for example, using reflective listening to help them process their thoughts and feelings. Here again we emphatically discourage the imposition of a belief-based therapeutic paradigm adopted by researchers and clinicians onto patients or study participants (see Moreira-Almeida et al., 2016; Koenig et al., 2020; Yaden et al., in press).

## Psychoanalytic and Psychodynamic

Psychedelics were generally not commented upon by the founders of the psychoanalytic movement (Sigmund Freud etc.—although Jung has a brief letter on this topic, see Jaffe, 2015), so the typical strategy of referencing and interpreting historical texts that often occurs in psychoanalytic circles is not as possible in this case. In general, psychoanalytic approaches postulate the existence of active unconscious forces or dynamics. Some contemporary researchers and clinicians have promoted the value of the psychoanalytic perspective in understanding psychedelic experience. For example, Carhart-Harris et al. (2014), claim that “scientific research with psychedelics has considerable potential for developing aspects of psychoanalytic theory.” Psychedelics are sometimes thought to reveal primary processes (unconscious functioning) in the same way that dreams do, which can then be interpreted by the analyst. Carhart-Harris et al. (2014) also quote Grof in saying: “The phenomenology of the psychodynamic experiences in LSD sessions is to a large extent in agreement with the basic concepts of classical psychoanalysis… Observations from LSD psychotherapy could be considered laboratory proof of the basic Freudian premises” (Grof, 1982).

Psychodynamic approaches generally involve less specific unconscious processes than psychoanalysis and refer to a wider range and more eclectic set of approaches than psychoanalysis (Wells, 1963; Eagle, 1984). Many forms of psychodynamic psychotherapy are commonly practiced in contemporary settings, and although their quality is highly variable, there is evidence for the effectiveness of many such approaches (Leichsenring and Steinert, 2017). In terms of psychedelic applications, the most prominent psychodynamic approach is that promoted by Grof (1977, 1980, 1982), which claims that the acute subjective effects of psychedelic substances can best be understood as a figurative and perhaps literal memory of being born (a view with Freudian roots). This “peri-natal theory” of psychedelic experience came to inform his preferred psychotherapeutic framing of psychedelic treatments and was highly influential in underground (i.e., illegal) psychedelic psychotherapy contexts.

At the present time, psychodynamic theory may be the most commonly utilized theory utilized by therapists conducting psychedelic psychotherapy, perhaps because it was ascendant at the time psychedelic therapy was developed and before research essentially stopped in the 1970s.

Furthermore, contemporary psychodynamic approaches conceptualize psychopathology in developmental, cultural, and temporal contexts in which a “persistent personality” navigates conflict and struggles via emotion-laden psychological defenses—understanding these dynamics is ultimately in the service of behavioral change (Fulmer, 2018). These defense mechanisms have been defined as “mental processes that operate unconsciously to reduce some painful emotion” (Paulhus et al., 1997, p. 543). This conceptualization may have been/be useful in approaching psychedelic experience, especially given the flexibility that this conceptualization provides and the intuitive nature of working with an “unconscious.” While sharing a context and goal with psychodynamic approaches, rather than unconscious processes, CBTs target empirically derived processes which are linked (through empirical evidence) to outcomes. As psychedelic therapy emerges from this period of relative quiescence, some have advocated for psychodynamic/psychoanalytic approaches to continue (see Harris, 2021). Psychedelics certainly offer interesting psychological content to try to understand using these perspectives.

However, there are reasons to question this approach. First, psychoanalytic/psychodynamic approaches have fallen largely out of synch with psychological research and cognitive science in general over the past several decades. Psychoanalytic/psychodynamic approaches were criticized decades ago as failing to keep pace with empirical research (e.g., Eysenck and Wilson, 1973; Beck, 1979). Psychoanalytic/psychodynamic approaches are largely separate from scientific research in general, and were used as a paradigm example of an unfalsifiable form of pseudoscience (Popper, 1983). For example, it is generally agreed that there is no way to falsify through a test the proposition of the id/ego/superego structure of the mind. Psychoanalytic/psychodynamic forms of therapy have been generally surpassed by cognitive approaches in terms of empirical support (Beck and Beck, 2011; Beck, 2019), which is discussed in the next section.

## Cognitive-Behavioral Approaches

The cognitive revolution in psychology built on earlier established empirically based behavioral principles and marked a shift away from the unfalsifiable psychoanalytic understandings of the mind (Miller, 2003). The most prominent pioneer of CBT was psychiatrist Aaron T. Beck, who de-emphasized unfalsifiable theories involving birth memories, early sexual conflicts, and supposed structures of the psyche. Instead, Beck’s view took a more empirical approach to psychotherapy development and treatment, focusing more on observable and reportable processes such as beliefs and emotions that could be empirically studied, in theory. In response to critiques that the cognitive approach is too superficial, Beck (2019, p. 17) famously said: “There’s more to the surface than meets the eye.” By this, Beck appears to mean that there are plenty of reportable beliefs, interpretations, emotions, and behaviors to work with in a psychotherapeutic setting without needing to postulate additional unconscious processes and forces.

Cognitive-behavioral approaches (including traditional CBT, DBT, and ACT, described below) are considered gold-standard forms of evidence-based psychotherapy for many psychological disorders by the American Psychological Association (APA) due to the substantial evidence supporting their efficacy (APA Presidential Task Force on Evidence-Based Practice, 2006; David et al., 2018). Over time, CBT has become more specifically described, articulated, and adapted to various populations and disorders.

Of the cognitive-behavioral approaches, traditional cognitive-behavioral therapy (CBT) involves a systematic assessment of thinking and behavior related to dysfunction and then intentional action is taken to help the client learn more adaptive thoughts and behaviors. Typically, clients are asked to fill out assessment measures specific to their presenting problems, and to self-monitor their own experience; therapists form their case conceptualizations based on these data (Persons, 2008). Sessions are structured to promote efficiency, and clients are guided by therapists to collaboratively evaluate and question their thoughts and beliefs (McGinn and Sanderson, 2001). There are many approaches within CBT to teach adaptive behavior which are both person- and pathology-specific. This traditional CBT approach has empirical support for its utility in treating a wide range of psychological disorders (APA Presidential Task Force on Evidence-Based Practice, 2006; David et al., 2018).

More recent versions of cognitive-behavioral approaches (such as DBT and ACT, described below) are often referred to as “third-wave” cognitive behavioral therapies (Hayes and Hofmann, 2017). Hayes and Hoffman highlight this third wave of cognitive-behavioral approaches as “a set of new behavioral and cognitive approaches… Third wave methods emphasized such issues as mindfulness, emotions, acceptance, the relationship, values, goals, and meta-cognition” (p. 245).

One widely practiced third-wave therapy is dialectical behavior therapy (DBT) created by Linehan (2020). It is now used to target a variety of mental health disorders where emotional dysregulation features prominently (Ritschel et al., 2018). DBT elaborates on traditional CBT in a number of ways. First is the central importance of mindfulness skills, which is one of four skills modules (the others are distress tolerance, emotion regulation, and interpersonal effectiveness; Rathus and Miller, 2015). Second, DBT has both an individual therapy and group component which work together to promote symptom reduction and skills use (Linehan, 2015). Third, DBT asks clients to call their individual therapists in crisis situations in order to be coached through effective skills use (*phone coaching*; Oliveira and Rizvi, 2018). These strategies are intended to teach adaptive behavior and ensure that it generalizes to situations in which it is most needed.

Another third-wave therapy is Acceptance and Commitment Therapy (ACT; pronounced “act”) the development of which was led by Steven Hayes. Like traditional CBT and DBT, in ACT there is an emphasis on developing awareness of thoughts, feelings, and sensations (Harris, 2006). Like DBT, ACT incorporates mindfulness techniques and promotes acceptance, however, unlike these approaches, ACT doesn’t directly target the reduction of dysfunctional thinking or difficult emotions, postulating instead that efforts to control or avoid these experiences contribute to suffering. The ACT approach targets six processes that promote *psychological flexibility*, defined as “contacting the present moment as a conscious human being, fully…and persisting with or changing a behavior in the service of chosen values” (Hayes et al., 2012, p. 96–97).

Finally, there are several notable ways cognitive-behavioral approaches may benefit from the partnering with psychedelic administration. First, psychedelics have an impact on processes, notably psychological flexibility (Close et al., 2020; Davis et al., 2020a) and outcomes (e.g., depression and anxiety, Davis et al., 2021; suicidal ideation; Zeifman et al., 2020) explicitly targeted by cognitive-behavioral approaches. Therefore, empirically understanding the psychedelic experience may provide insight into cognitive-behavioral approaches (and vice versa). This is exemplified by recent work exploring the overlap between psychedelic experience and the sense of self in ACT (Hayes et al., 2020). The authors make explicit that this overlap is an opportunity both for ACT to guide future research in psychedelic science *and* “learn more about flexibility processes” (p. 36). Second, nesting psychedelic administration in cognitive-behavioral-based preparation and integration sessions may amplify the therapeutic effects (and generalization) of these processes and outcomes. Ultimately, consistent with the scientific values of cognitive-behavioral approaches, these sorts of potential synergies must be explicitly tested.

Taken together, traditional CBT, DBT, and ACT (we refer to these three together as cognitive-behavioral approaches) have the merits of more empirically testable claims, theoretical assumptions more linked to contemporary psychological science, and a large base of empirical support for their safety and efficacy. We therefore believe these cognitive approaches ought to be the default psychotherapeutic paradigm paired with psychedelic treatments.

## Addressing Objections to the Cognitive-Behavioral Approach

We have encountered some resistance to the view that cognitive-behavioral approaches (CBT, DBT, and ACT) should be the default approach to psychedelic psychotherapy in contemporary healthcare and research settings. Some common objections to this view include issues related to (1) the high prevalence of participants’ reports of religious/spiritual/unconscious material, which do not feature prominently in cognitive-behavioral approaches (2) lack of studies pairing CBT with psychedelics, (3) concerns that cognitive-behavioral approaches are often rigidly manualized treatments that unduly restrict patient and clinician choice; and (4) unfamiliarity with concepts from cognitive-behavioral approaches that are relevant to psychedelic treatments.

Regarding objection one, the prevalence of participant reports of content related to religious, spiritual, and unconscious processes, we admit that such reports are prevalent and important to acknowledge. We reiterate our view that participants and patients are free to bring *their own* beliefs and ideologies into psychedelic treatments–as should be the case in all medical and psychotherapeutic treatments (see Peteet et al., 2011). In other words, we are *not* commenting on the frame that participants and patients ought to bring, but rather that used by researchers/clinicians (see Johnson, 2020). In addition, there is much writing to guide how spiritual/religious content can be incorporated into CBT treatments (e.g., Nieuwsma et al., 2016) and ACT, specifically, has a robust theory that addresses typical spiritual experiences that occur in psychedelic-assisted therapy (Luoma et al., 2019) such as mystical experiences that involve self-transcendence (Yaden et al., 2017a) or feelings of interconnection with others or the universe (Watts and Luoma, 2020).

Regarding objection two, the lack of studies pairing CBT with psychedelics: The objection is sometimes made that because psychedelic treatments are so novel, there is a paucity of research on all psychotherapeutic pairings—and, therefore, they should *all* be tried and no particular approach should be assumed the default. While we agree that research is on-going and relevant approaches should be tested, we do not agree that all approaches are equally reasonable candidates. We argue that we have good reasons to choose approaches that fit best with contemporary scientific research, are suited to secular treatment contexts, carry less risk of being culturally offensive, and have more evidence of safety and effectiveness. We believe that CBT represents the strongest family of approaches in each of these regards. Lastly, and crucially, *there have already been successful pairings of cognitive-behavioral approaches with psychedelic treatments*. Specifically, Johnson et al. (2014) combined traditional CBT with psilocybin in a tobacco use disorder trial. Also, ACT has been combined with psilocybin in the treatment of depression (Carhart-Harris et al., 2016; Sloshower et al., 2020).

Regarding objection three, that cognitive-behavioral approaches leads to overly restrictive manualized treatment, we wish to emphasize that we are *not* advocating for the strict application of a particular manualized process in each psychedelic study/treatment, nor for particular interventions to be used in specific sessions. The idea that CBT is an approach that is inherently restrictive of clinician flexibility, creativity, and responsiveness is a straw man. Of course, cognitive-behavioral approaches will need to be adapted to the context of use, for example alongside psychedelic substances (there are numerous examples of doing this for particular diagnoses, patient populations, and other contextual factors; e.g., see Wenzel et al., 2012). Furthermore, any approach can be rigidly applied, including non-cognitive-behavioral approaches. In summary, we believe that cognitive-behavioral approaches should not be used without adaptation to this unique therapeutic context and to the individual patient/participant, but this concern applies to other theoretical approaches as well.

Regarding objection four, unfamiliarity with concepts from cognitive-behavioral approaches that are relevant to psychedelic treatments, we acknowledge that not all researchers and clinicians have had exposure to cognitive-behavioral approaches (e.g., CBT, DBT, ACT) and particularly how cognitive-behavioral approaches are capable of addressing the unique characteristics involved in psychedelic assisted psychotherapy, such as spiritual experiences (see Luoma et al., 2020). Furthermore, we recognize that there are a great number of popular books and articles advocating for the pairing of psychedelic treatments with indigenous practices, new age spirituality, and psychodynamic approaches—-and that there is a relative paucity of such resources for cognitive-behavioral approaches in the domain of psychedelic treatments. This simply speaks to the need for more work to disseminate cognitive-behavioral approaches that address issues which commonly occur during psychedelic states. One advantage of utilizing cognitive-behavioral approaches with psychedelic administration is that there is a long tradition and much expertise in learning how to rigorously adapt and test cognitive-behavioral principles in a wide variety of clinical contexts.

To be clear, our view that cognitive-behavioral approaches should be considered default for psychedelic treatments rests upon the context in which psychedelic administration is being delivered. We do not posit that all psychedelic use everywhere should be grounded in cognitive-behavioral approaches. However, in the current clinical research context, psychedelic-psychotherapy research programs are targeting outcomes for which cognitive-behavioral approaches have been shown to be effective for in experimental studies (e.g., depression and anxiety, Davis et al., 2021; suicidal ideation, Zeifman et al., 2020). Not only are cognitive-behavioral approaches effective for these outcomes, but they are also currently the gold standard of evidence-based care (APA Presidential Task Force on Evidence-Based Practice, 2006; David et al., 2018). Reiterating the synergy mentioned above regarding the overlap between the effects of psychedelic experience and processes and outcomes targeted in cognitive-behavioral approaches, these approaches are the best fit empirically and ethically.

The next section represents an overview of several concepts and techniques from cognitive-behavioral approaches that appear highly relevant to psychedelic psychotherapy (see Table 1).

**TABLE 1:** Concepts from cognitive-behavioral approaches relevant to psychedelic treatments, by therapy phase (preparation, dosing session, integration).

Concept	Citations	Description	Relevance to psychedelic treatments
**Preparation**			
**CBT**			
*Structured session format*	McGinn and Sanderson, 2001	Predictable session structure (check-in, setting agenda, completing agenda, summary and assigning homework/action plan).	Make efficient use of time, provide structure and predictability for participants, encourage collaboration and rapport.
*Psychoeducation*	McGinn and Sanderson, 2001	Summary of initial assessment results (discussion of presenting problem/diagnosis), orienting clients toward the treatment modality and providing a rationale for treatment.	Psychoeducation for psychedelic therapy should communicate how psychedelic therapy works or that the mechanism is hypothetical if still under investigation.
*Self-monitoring*	Egan et al., 2014	Encourage clients to pay attention to thoughts, emotions, and behaviors.	Empowers participants to develop a sense of empiricism about their own experience, develop a sense of baseline experience.

**Preparation:** **DBT**			
*Pre-treatment and Commitment strategies*	Swenson, 2016	Sessions are aimed at increasing commitment to the treatment plan and motivating engagement in therapy.	For the practitioner/monitor: reinforces that treatment is ultimately the participant’s decision and facilitates space for that decision to be explored even once “treatment” has begun.
*Therapy-Interfering Behavior (TIB) as a key target*	Linehan, 1993, p. 129	Focus on behaviors or patterns of interaction that could interfere with effective therapy.	Allows for an open conversation about which parameters might be therapy interfering for given client, session monitors/practitioners become mindful of their own potentially therapy-interfering behaviors
*Skills training*	Linehan, 1993, p. 329	Teach patients skills to address difficult thoughts and emotions.	Provide participants with tools to aid in tolerating difficulties or making changes in their lives even before any drug is administered. Skills can be called upon during the session and integration phases.

**Preparation:** **ACT**			
*Psychological flexibility*	Luoma et al., 2017	Exercises aimed at supporting the three pillars of psychological flexibility–openness, awareness, and engagement to help clients respond effectively to the challenges of life.	Exercises based on openness, awareness, and engagement could conceivably potentiate psychedelic sessions.
*Developing alternatives to struggle and avoidance*	Bennett and Oliver, 2019	Help the client be more open to new patterns of behavior which are not organized around avoidance and escape; cultivate openness and acceptance	Acceptance has been proposed by previous authors as one process through which psychedelics may have their effects (Watts et al., 2017). Practice with this orientation may be useful during session as well.
*Connecting with values*	Luoma et al., 2017, p. 29	Clarification of values and consideration of the extent to which current life aligns with values.	Psychedelic therapy has been reported to result in shifts in people’s life priorities (Belser et al., 2017; Swift et al., 2017) and increase connection with core values (Noorani et al., 2018). Clarification and discussion of values in prep may later facilitate integration.

**Dosing session**			
**CBT**			
*Core beliefs and cognitive distortions*	Beck and Haigh, 2014	Beliefs and thoughts that address the self, one’s future, and the world.	During dosing sessions, a participant may encounter core beliefs and cognitive distortions.
*Cognitive restructuring*	Beck and Haigh, 2014	Targeting dysfunctional or biased reasoning (including core beliefs and cognitive distortions) and to help clients evaluate them.	There is initial evidence to suggest that psychedelic therapy can change various beliefs. Training with this skill may facilitate this desired outcomes.
*Relaxation techniques*	Clark and Beck, 2010	These techniques include *progressive muscle relaxation (PMR*, *applied relaxation*, and *breathing retraining.*	If these are practiced in advance, session monitors could prompt clients to use techniques (functionally similar to therapeutic touch) to restore a sense of safety and empower participants to continue with the session, should anxiety or panic occur.

**Dosing session:** **DBT**			
*Mindfulness skills*	Linehan, 2015	The core mindfulness skills are the *what* (e.g., observe, describe, and participate) and *how* skills (e.g., non-judgmentally, one-mindfully, and do what works)	Training in mindfulness skills taught during preparation may help client to experience the session in a more engaged manner.
*Emotion regulation skills*	Linehan, 2015	Emotion regulation skills are often taught in DBT with the caveat that we cannot have total control over our emotions, but useful for modulating emotion.	In session, participants may be better to able to articulate and manage what emotions are coming up and thereby give session monitors a better sense of when to intervene and minimize unnecessary disruption
*Distress tolerance skills*	Linehan, 2015	*Crisis survival skills* (such as the relaxation techniques described in traditional CBT) and *reality acceptance skills*, which promote a conscious commitment to accept situations beyond one’s control.	When challenging experiences arise in the session phase, participants can be encouraged to use the *Turning the Mind* skill, which is a stance cultivated through practice involving choosing to accept one’s present experience.

**Dosing session:** **ACT**			
*Defusion*	Luoma et al., 2017, p. 99	Exercises and discussion to help participants to get a better sense of the nature of their unique process of thinking rather than getting caught up (or fused) with a particular thought, sensation, image, or memory.	May help clients be able to let go of the struggle with attempting to understand or more make sense of the psychedelic experience in the moment, to help them engage more fully therapy.
*Acceptance*	Hayes et al., 2012	Allow thoughts and feelings to come and go without trying to change them.	Helpful for navigating challenging experiences. Participants could be cued to engage in acceptance during difficult moments.
*Present moment awareness*	Harris, 2009, p. 156	Involves paying attention to one’s moment by moment experience (internally and externally)	Helpful for clients who get caught up in repetitive thinking, catastrophic worry, or otherwise unable to return to the psychedelic experience.

**Integration**			
**CBT**			
*Teaching adaptive behavior and goal setting*	McGinn and Sanderson, 2001	Traditional CBT includes strategies to set specific goals around desired ends and tracking progress.	Integrate the discovery and motivation from the dosing session phase into more lasting behavioral change through setting specific and attainable goals.
*Setting homework or action plans (e.g., behavioral experiments)*	Bennett-Levy et al., 2004	Client and session monitor activities client can do during the week to practice new behaviors and/or test thoughts and beliefs.	May help to carry over insights from the “non-ordinary” experience in the dosing session to one’s return to “ordinary” life and help to form new habits, ways of interacting with the world
*Monitoring Progress*	Lambert et al., 2003	Systematic assessment, through validated measures, throughout course of treatment.	Ongoing psychometric assessment to supplement clients’ reports can help to assess progress see what strategies and behaviors are most helpful in facilitating desired change.

**Integration:** **DBT**			
*Diary cards*	Linehan, 1999	Track behavioral targets, emotions, and skill use over the previous week.	Monitor ongoing challenges, successes, and progress toward goals.
*Chain analysis*	Rizvi and Ritschel, 2014	Visually depicting the sequence of events (both internal and external) that led up to a target behavior, as well as consequences.	May be used to understand important or profound moments that participants experience in their daily lives and identify opportunities for intervention or new ways of responding.
*Cultivating a dialectical stance*	Rathus and Miller, 2015	(1) Working on acceptance through validation, (2) working on change through behavior change, and (3) synthesizing these approaches in an adaptive manner.	The dialectic between acceptance and change may have come up in the psychedelic experiences, which can be discussed.

**Integration:** **ACT**			
*Metaphor and experiential exercises*	Bennett and Oliver, 2019	Two clinical tools that are frequently used and allow clients to learn from direct experience or experiential language.	The use of metaphor and experiential exercises is a way of helping to integrate an experience that is difficult to describe in words using therapeutic approaches that are also meant to go beyond words.
*Self-as-context*	Luoma et al., 2017, p. 28	Practice with the concept of “A continuous and secure ‘I’ from which events are experienced, a self that contains but is also distinct from those events.”	An observing sense of self can provide a stable place from which to observe and process the alterations in sense of self and other that can occur during psychedelic sessions.
*Committed action*	Hayes et al., 2012, p. 328	Clients commit to specific actions in their lives that will help clients align their daily activities with their values.	This concept (and change process) is of great value in psychedelic therapy, to facilitate lasting behavior change as a result of the sometimes-profound experiences had during psychedelic sessions.

*For each of the three phases of psychedelic-assisted psychotherapy, Preparation, Dosing Session (“Session”), and Integration, three concepts from each of the three cognitive behavioral therapies, CBT, DBT, and ACT, were identified as relevant. Together, these 27 distinct concepts are not meant to be an exhaustive list, but rather depict the suitability of the cognitive behavioral therapy framework as the default for psychedelic-assisted psychotherapy.*

## Concepts From Cognitive Behavioral Therapy Relevant to Psychedelic Treatments

There are a number of concepts from cognitive-behavioral approaches that appear to be highly relevant to psychedelic treatments. In this section, we provide concepts from cognitive-behavioral approaches to inform each step of psychedelic treatments, which can usefully be divided into (1) preparation, (2) dosing sessions, and (3) integration. In the following, we describe these three broad stages of this process (as described in, for example, Johnson et al., 2008, 2019) and then list concepts from CBT, DBT, and ACT that are relevant with a brief explanation of each. Again, this is not meant to be a comprehensive list—and there is overlap in concepts across CBT/DBT/ACT (i.e., each concept is not necessarily unique to each framework), so this should be considered a starting place to show the rich set of concepts to draw from in these psychotherapeutic paradigms. Note that we use the terms patients (but the terms clients and participants can also be used interchangeably) and therapist (but the terms guides, monitors, facilitators, and clinicians can also be used interchangeably).

### Preparation

Preparation consists of the sessions that occur in the days and weeks prior to administration of the psychedelic, during which time participants become familiar with the facilitators who will be present during their dosing sessions. This stage often includes extensive psychoeducation about the framework of the dosing sessions, the effects of the substance in question, and experiences likely to occur during the dosing session. Elements related to various theories of intervention may be brought into this stage as well to help orient patients toward the dosing session and to prepare for any difficulties that may arise. (Various expectancies may also be introduced—inadvertently or intentionally—a topic of on-going empirical research). Below we describe how cognitive-behavioral approaches might be used during preparation sessions.

It is commonly accepted across nearly all psychedelic-assisted therapy approaches, including cognitive-behavioral approaches, that a collaborative therapeutic alliance is essential. This alliance involves having shared goals, an understanding of each other’s roles, and a degree of comfort working together (Egan et al., 2014). This alliance helps establish a sense of safety and trust in the therapeutic context that is thought to be important in facilitating an effective psychedelic experience. Cognitive-behavioral approaches generally view a solid therapeutic alliance as *necessary-but-not-sufficient* (Beck et al., 1979), and thereby includes other strategies often used in preparing and orienting clients to therapy.

### Cognitive Behavioral Therapy

#### Structured Session Format

A hallmark of traditional CBT sessions is the predictable structure of the session, which is itself a therapeutic tool. Sessions typically have four components: (1) initial check-in, (2) setting an agenda for the session, (3) completing the agenda, and (4) summarization and setting action plans (McGinn and Sanderson, 2001). Examples of agenda items include: treatment targets occurring both in and out of session, high priority-problems or goals, and targets the client wants to put on the agenda (Persons, 2008). Setting the agenda, like the rest of CBT, is a *collaborative* process—the client and therapist are working as a team (Persons, 2008).

The structure of a session provides both patients and therapists with a sense of what to expect. Psychedelic psychotherapy sessions that are predictable in form can help session monitors to make efficient use of time as there is limited time in any therapy session. Organizing and structuring time provides scaffolding for participants and communicates to them that the therapist respects their time and wishes to make the session maximally useful for them. This, along with the predictability and familiarity, can encourage rapport between session therapists and patients.

#### Psychoeducation

Psychoeducation is a key aspect of traditional CBT, DBT, and ACT. CBT psychoeducation includes a summary of initial assessment results, orienting patients toward the treatment modality and providing a rationale for interventions or treatment strategies (McGinn and Sanderson, 2001). For instance, in psychoeducation for obsessive-compulsive disorder, a patient receives didactic instruction on the cycle of avoidance that maintains unwanted intrusive thoughts and how therapy, using this understanding, is expected to target these symptoms (Abramowitz and Jacoby, 2015). This normalizes symptoms and provides a rationale for why the proposed treatment is expected to be clinically useful.

Psychoeducation for psychedelic therapy, for instance, might involve education about the patient’s symptoms and what the treatment itself will entail. It is important that psychedelic psychotherapy psychoeducation also address how psychedelic psychotherapy is expected to target a participant’s symptoms. If these mechanisms are unknown, hypothetical or under empirical investigation, then *that* should be communicated transparently to the patient during psychoeducation sessions as well as during the informed consent process (Smith and Sisti, 2021).

#### Self-Monitoring

Self-monitoring is a skill taught to clients early in CBT, that aims “to train clients to pay attention to or monitor particular cognitions, emotions, and or behavior” (Egan et al., 2014, p. 137). Each week during the initial check in and homework review, the therapist can point out patterns and highlight the ways in which these emotions, thoughts, and behavior are affecting functioning.

Self-monitoring could be relevant to psychedelic psychotherapy because it empowers participants to develop a sense of empiricism about their own experience. By encouraging the patient to self-monitor prior to drug administration, it can help to meaningfully develop a sense of baseline experience. Over time, patients can compare their current responses to earlier sessions to see for themselves how treatment is going using online surveys or smart-phone based experience sampling methods (Insel, 2017).

### Dialectical Behavior Therapy

#### Pre-treatment and Commitment Strategies

DBT progresses through various of stages and begins with a series of sessions referred to as *pre-treatment* which are aimed at increasing commitment to the treatment plan and motivation to engage in therapy (Swenson, 2016). Linehan (1993) remarks that “people are more likely to do what they agree to do” (p. 284). An example of a commitment strategy is *door-in-the-face* technique, which asks for a large commitment to change a behavior with the aim of getting any smaller commitment from the patient (Swenson, 2016).

Building commitment in psychedelic psychotherapy preparation sessions may be useful for both the participant and session monitors. Commitment strategies involve conversations around motivations for seeking therapy. It is useful for the session monitor because it reiterates the stance that treatment is ultimately the participant’s decision and facilitates space for that decision to be explored even though “treatment” has begun (this can be similar to motivational interviewing techniques, discussed later). If commitment is built, this commitment can also be referred to and re-established throughout the course of psychedelic psychotherapy and perhaps enhance study retention.

#### Therapy-Interfering Behavior as a Key Target

In DBT, treatment targets are prioritized. In initial sessions following pre-treatment (i.e., Stage 1), the first target is suicidal or life-threatening behavior and the second is therapy-interfering behavior (TIB; Swenson, 2016). TIBs are behaviors by “both the client and therapist that interfere with effective therapy” (Linehan, 1993, p. 129). Examples include a client’s non-attendance or burnout on the part of the therapist (Chapman and Rosenthal, 2016). By prioritizing TIB in this way it promotes case conceptualizations that uphold a client’s meaningful contact with treatment as crucial.

TIBs is an element of DBT that doesn’t fit neatly into one phase of psychedelic psychotherapy (as is the case with many of these concepts). Preparation provides an opportunity to discuss expectations and parameters for what might occur during dosing sessions. For example, in dosing sessions, there is an emphasis on session monitors remaining less involved, redirecting participants toward their own experience, and lending a hand to hold if asked. By incorporating TIB into preparation for psychedelic therapy, it allows for an open conversation about whether these parameters might be therapy-interfering for a given client. Additionally, session monitors become mindful of their own potentially therapy-interfering behaviors, say, if a monitor is more inclined to reach out with a hand to hold for a given client before being asked.

#### Skills Training

Skills training is a very broad category and can be thought of as an element of all cognitive behavioral approaches. There are several possible DBT skills to draw from, which are covered under the dosing session section, but here we offer discussion of what could be covered in preparation. The DBT skills for adults consist of four modules: mindfulness, distress tolerance, emotion regulation, and interpersonal effectiveness (Rathus and Miller, 2015). There is empirical support for DBT skills training as a standalone treatment for various psychopathologies (Valentine et al., 2014).

Psychedelic psychotherapy could benefit from incorporating select DBT skills training into preparation sessions for two broad reasons. First, these skills provide participants with tools to aid in tolerating difficulties or making changes in their lives even before any drug is administered. Second, these skills can be called upon during the dosing session and integration phases and strengthened so that participants develop a proficiency in these skills that gets them closer to the life they want to be living—in DBT referred to as *a life worth living* (Swenson, 2016).

### Acceptance and Commitment Therapy

#### Psychological Flexibility

The overarching goal of ACT is the development of psychological flexibility, a capacity to respond effectively to the challenges of life in an ongoing way. Rigidity and inflexibility are believed to be at the heart of psychopathology (e.g., Luoma et al., 2017; Wolff et al., 2020). In this approach, clients are invited to reflect on and be guided by values-based treatment goals, which do not involve targeting the cessation or reduction of difficult thoughts or feelings (Hayes et al., 2012).

Psychological flexibility may be helpful in framing how dosing sessions are approached and may also be consistent with emerging evidence. A psychological flexibility model de-emphasizes attempts to try rid oneself of unpleasant experiences (*experiential avoidance)*, something that is unlikely to be successful during dosing sessions, and instead emphasizes the utility of openly embracing all the experiences of life in attempt to learn what they have to say about how to live well. Some studies have shown that psychological flexibility improves during and after therapeutic psychedelic experiences (Davis et al., 2020a; Zeifman et al., 2020) and is associated with therapeutic outcomes. Below we outline how work aimed at supporting the three pillars of psychological flexibility—openness, awareness, and engagement—could conceivably potentiate psychedelic sessions.

#### Developing Alternatives to Struggle and Avoidance

Most clients come to therapy with the hope that therapy will rid them of painful emotions and thoughts, but unfortunately rigid attachment to such avoidance can promote suffering, as avoidance is central to many forms of pathology. ACT begins to address this avoidance by helping clients to examine the workability of their attempts to avoid or control challenging emotions and thoughts, with the goal of helping the client be more open to new patterns of behavior not organized around avoidance and escape (Bennett and Oliver, 2019). ACT directly encourages acceptance as an alternative and offers various metaphors and exercises as ways to build this ability to let go of struggling with difficult experiences. For example, the experiential *Tug of War* exercise involves the client and therapist engaging in an actual tug of war with the therapist representing the clients’ challenging thoughts, emotions and sensations (Bennett and Oliver, 2019, p. 131–133). The exercise ends with the acknowledgment that instead of struggling, clients can always “drop the rope” (Bennett and Oliver, 2019, p. 133).

In preparation sessions, it may be advantageous to cultivate this *openness to acceptance* and the idea that attempting to control thoughts and feelings often creates suffering. This seems especially relevant to psychedelic psychotherapy as acceptance has been proposed by previous authors as one process through which psychedelics may have their effects (Watts et al., 2017) and thus an explicit focus on fostering and supporting this process may fit particularly well with the psychedelic experience.

#### Connecting With Values

In ACT, *values* refer to “chosen qualities of actions that can never be obtained as an object but can be instantiated moment by moment in actions of being and doing” (Luoma et al., 2017, p. 29). Values are more like the “compass heading” (Bennett and Oliver, 2019, p. 209) or the direction for life, rather than the destination. Questions that are sometimes used to help clients identify their values include, “What kind of mother/son/neighbor/citizen/worker do I want to be?” Getting clients to connect with values offers them an opportunity to create meaning in their lives, right away, in each action they take (Harris, 2009).

Psychedelic therapy has been reported to result in shifts in people’s life priorities (Belser et al., 2017; Swift et al., 2017) and increase connection with core values (Noorani et al., 2018). ACT provides a way to frame these shifts in values, a means to resolve any values conflicts that might arise as priorities shift, and support in bridging these experiences toward meaningful life changes. In addition, work on values during preparation could help clients identify an intention for dosing sessions that is self-chosen and hence less likely to avoid patterns of avoidance that maintain suffering.

### Psychedelic Administration Session

The psychedelic administration session (or dosing session) is the period of time during which the psychedelic is administered and the acute subjective effects are experienced. Typically, participants will lie down on a couch with eyeshades and headphones in order to be as comfortable as possible during their experience (these are parameters that are being researched in ongoing studies; see Johnson et al., 2008, for a thorough description and safety considerations). There are generally two monitors in the room at all times and the sessions are unobtrusively recorded all measures for the safety of participants and patients. Participants may talk with the monitors, but in such cases, monitors might encourage participants to instead attend to their own inner experience. Participants can, at some research centers such as at Johns Hopkins, ask for the facilitator to hold their hand otherwise offer some sort of minimal supportive touch if frightened or anxious. The following are concepts or skills from cognitive-behavioral approaches that may be relevant during the psychedelic administration session.

### Cognitive Behavioral Therapy

#### Core Beliefs and Unhelpful Thoughts

Through psychoeducation and self-monitoring, CBT clients become familiar with their core beliefs and unhelpful thoughts. These core beliefs often manifest as automatic thoughts (McGinn and Sanderson, 2001). An example of a core belief is: “I am unlovable.” *Unhelpful thoughts* are predictable and systematic forms of maladaptive thinking (Yurica and DiTomasso, 2005). Becoming aware of one’s unhelpful thoughts comprises an important part of CBT.

During dosing sessions, a participant is likely to encounter core beliefs and unhelpful thoughts because this content, in many cases, is so automatic and engrained. The psychedelic experience offers a new mode by which one may be more likely to identify and engage with them due to the new perspectives introduced during the acute subjective effects. By encouraging participants to discover and label their own automatic thoughts, they may be primed to encounter and discover insights about them in session. Also, by encouraging participants to discover and label their unhelpful thoughts in prep, participants may develop a conceptual scaffolding to use when encountering these unhelpful through in session.

#### Cognitive Restructuring

Cognitive restructuring in CBT refers to targeting dysfunctional thoughts and helping clients evaluate them (Beck and Haigh, 2014). McGinn and Sanderson (2001) describe cognitive restructuring as a process where “clients are trained to increase awareness of ongoing ‘stream of consciousness’ during episodes of increased affect, exposing these rigid ‘automatic thoughts’ which accompany emotional responses” (p. 29).

The concept of cognitive restructuring may be relevant to psychedelic psychotherapy because there is initial evidence to suggest that psychedelic therapy can change beliefs (Nayak et al., in preparation^1^; Timmermann et al., 2021). Cognitive restructuring (with its necessary component of self-monitoring) offers participants an empirically rooted system to use to monitor, discover, label, evaluate, and test thoughts and beliefs. Therefore, during the dosing session phase, session monitors could gently empower participants to use this system as they see fit to navigate their experience. While more active or structured interventions such as this have generally not been included in dosing sessions in current clinical trials, it provides an interesting potential intervention to explore in future research, if able to be adapted to the context of a dosing session. There exists a tradition, often termed psycholytic therapy (e.g., see Garcia-Romeu and Richards, 2018 for a brief description), of using more active psychoanalytic techniques such as interpretation during psychedelic states. Our suggestion is to consider broadening this strategy of utilizing more active interventions during psychedelic states by testing more recent and empirically based strategies.

#### Relaxation Techniques

Relaxation Techniques (*distress tolerance skills* in DBT) are sometimes used in traditional CBT. These techniques include *progressive muscle relaxation (PMR)*, which involves tensing and relaxing specific muscle groups, *applied relaxation*, similar to PMR but paired with cues (e.g., “relax”) and applied outside of the session, and *breathing retraining*, which entails teaching diaphragmatic breathing (Clark and Beck, 2010).

Relaxation techniques are likely to be useful in psychedelic psychotherapy for similar reasons that they are useful in CBT. Anytime emotional or physiological arousal becomes therapy-interfering during the dosing session or otherwise, these relaxation techniques may help decrease arousal so that the participant can continue to engage in treatment. In psychedelic psychotherapy, should pre-session or in-session anxiety or panic occur, session monitors can use techniques (functionally equivalent to therapeutic touch) to restore a sense of safety and empower participants to continue with the session.

### Dialectical Behavior Therapy

#### Mindfulness Skills

In DBT, the mindfulness module aims to cultivate an awareness of internal and external present moment experience. The core mindfulness skills are the *what* (observe, describe, and participate) and *how* skills (non-judgmentally, one-mindfully, and do what works; Linehan, 2015). Rathus and Miller (2015) highlight that “these skills form the core of the entire skills set, as individuals need these skills to be able to make use of the other DBT skills” (p. 97).

During the dosing session phase, session monitors could encourage participants to call upon mindfulness skills taught during preparation. For instance, the words “mindfulness skills” could become a cue for clients to observe their experience, describe what they notice and participate in the present moment. This is the reason why skills training as a whole was suggested in the “preparation” section above, so that session monitors could cue these skills in session.

#### Emotion Regulation Skills

Emotion regulation skills are often taught in DBT with the caveat that we cannot have total control over our emotions (Linehan, 2015). Instead, these skills are useful in modulating emotion. Some targets of emotion regulation skills include understanding and naming emotions, changing emotional responses, reducing vulnerability to extreme emotions, and managing difficult emotion (Linehan, 2015).

In psychedelic psychotherapy, teaching participants to understand and name their emotions could create a sense of emotional literacy. In session, participants may be better to able to express what emotions are coming up and thereby give session monitors a better sense of when to intervene and minimize unnecessary disruption.

#### Distress Tolerance Skills

Distress tolerance skills involve more than just managing difficult emotion, rather, this module is for situations that are considered *crises* (Linehan, 1993). The distress tolerance module comprises two parts: *crisis survival skills* (such as the relaxation techniques described in traditional CBT) and *reality acceptance skills*, which promote a conscious commitment to accept situations beyond one’s control to minimize suffering though it may not “fix” the situation itself (Linehan, 2015).

During the dosing session, the reality acceptance skills in this module seem especially useful. When challenging experiences arise in the session, participants can be encouraged to use the stance cultivated through practice that acceptance is a choice one must make “over and over again” (Rathus and Miller, 2015. p. 151).

### Acceptance and Commitment Therapy

#### Defusion

Defusion refers to the idea that one’s identity does not consist of one’s passing thoughts. That is, one can look “*at* thoughts rather than *from* thoughts” (Luoma et al., 2017, p. 99). The aim of defusion is to reduce the influence of narrow and rigid cognitive forms of responding. Through metaphor and experiential exercises, clients come to learn that thoughts need not control behavior (Hayes et al., 2012). Having this distance from thoughts can liberate clients to move in valued directions.

Defusion could be of great utility in psychedelic psychotherapy by allowing patients to notice and disengage from repetitive or unproductive lines of thinking such as obsessive rumination or worry that might occur in session. It may also help clients be able to let go of the struggle with attempting to understand the sometimes confusing components of psychedelic experience that may interfere with full engagement in the therapy.

#### Acceptance

Experiential acceptance is the ability to allow thoughts and feelings to come and go without struggling against them or trying to change them. In ACT, acceptance is an action one can engage in as an alternative to escape, avoidance, or thought suppression (Hayes et al., 2012). Like DBT, in ACT acceptance is viewed as a process, and defined as “the voluntary adoption of an intentionally open, receptive, flexible, and non-judgmental posture with respect to moment-to-moment experience” (Hayes et al., 2012, p. 272).

Acceptance as it is construed in ACT could be useful to the dosing session phase in two ways. If, for example, the tug-of-war exercise were introduced during the preparation phase, then the cue “drop the rope” by a therapist might encourage participants to stop resisting challenging experiences that arise. Second, framing acceptance as a values-based choice empowers participants to choose to stay with the struggle rather than feeling coerced by the therapist or their own self-injunctions.

#### Present Moment Awareness

Defusion and acceptance promote an “open” response style, and present moment awareness promotes a “centered” one (Hayes et al., 2012). It is through contacting the present moment that clients contact a “firm foundation for awareness and action” (Hayes et al., 2012, p. 219).

Defusion and acceptance can promote an open stance toward challenging experiences that arise during psychedelic administration sessions and present moment awareness involves engaging with that experience (rather than being carried away by it or struggling against it). ACT techniques that foster *present moment awareness* might be helpful for clients who caught up in repetitive thinking, catastrophic worry, or otherwise unable to return to what there might be to learn from the psychedelic experience.

### Integration

Integration refers to the therapeutic support offered after the acute subjective effects subside, which can be scheduled in the hours, days, weeks, and months following the session. Integration typically involves participants and patients describing their experiences to a clinician, working to make sense of any confusing experiences. Integration also typically involves identifying whether there are any important implications from the dosing session for how the person might want to live their life going forward and considering how to put those implications into practice. There are a number of concepts from cognitive-behavioral approaches that clinicians could draw from during integration in order to help participants and patients understand and make sense of their experiences while leveraging them for therapeutic benefit.

### Cognitive Behavioral Therapy

#### Teaching Adaptive Behavior and Goal Setting

Traditional CBT includes strategies to teach adaptive behavior, such as problem-solving, pleasant activities scheduling, contingency procedures, skills training, and exposure (McGinn and Sanderson, 2001). CBT can involve setting behavioral goals toward valued ends. Participants and patients can then be reminded and supported in making measurable progress toward those goals using concepts like behavioral activation (e.g., Sturmey, 2009), which involves setting more proximate and attainable goals as steps toward larger goals. Behavioral activation may help individuals re-engage in activities that bring them a sense of mastery and pleasure by having them work toward these goals in a systematic way.

Teaching adaptive behavior in psychedelic psychotherapy is crucial because motivational urges or insights gained in the dosing session phase do not automatically impart ability or reduce barriers to engaging in adaptive behaviors. For example, a participant may discover that they are not satisfied by their career and have an urge to change. Also, scheduling pleasant activities to help them engage in what they find fulfilling can serve to integrate the discovery and motivation from the dosing session phase into more lasting behavioral change. There are any number of therapeutic goals that could be set during integration.

#### Assigning Homework: Behavioral Experiments

Behavioral experiments are a common form of homework aimed at testing the validity of and updating potentially erroneous or maladaptive beliefs. In these experiments, patients test out predictions such as, “She wouldn’t want to go to a movie with me,” by performing the behavior in question (inviting the friend to a movie) and seeing what actually results.

Homework, and in particular, behavioral experiments have potential value in psychedelic psychotherapy. This concept may help to carry over insights from the “non-ordinary” experience in the dosing session to one’s return to “ordinary” life. For example, if, during the psychedelic administration session, a participant has a profound sense that a particular difficult relationship needs tending to, a clinician could assign the homework of engaging in a behavioral experiment of actually tending to those difficult relationships and seeing what happens. The individual could then test whether their beliefs about a given difficult relationship holds true after the relationship has received additional time and attention paid to it.

#### Monitoring Progress

Monitoring progress through empirically validated measures is at the heart of CBT. There is evidence that when therapists monitor clients’ progress through assessment, clients experience better outcomes (Lambert et al., 2003). Specific measures are tailored to the client’s presenting symptoms and goals for treatment. Repeated measurement over time allows the therapist to adapt to the treatment to the clients’ response. For example, if a particular strategy aimed at improving sleep does not result in improved sleep, the therapist and client may decide to change course. Rather than being viewed as a nuisance, such measures, when used effectively, can be a helpful adjunct to the therapeutic process.

Ongoing psychometric assessment in psychedelic psychotherapy (e.g., using online survey links or smart-phone based experience sampling methods) could provide the clinician with a means through which to supplement clients’ narrative reports during therapy. It also allows clinicians to develop an empirically grounded case conceptualization, measuring specific constructs that may mediate change (e.g., psychological flexibility) along with outcome-based measures (e.g., scores of depression or anxiety). Furthermore, assessment helps to keep clinicians from “seeing” change that is not there.

### Dialectical Behavior Therapy

#### Diary Cards

In individual DBT sessions, participants turn in a *diary card*, which tracks life-threatening behaviors, as well as other behavioral targets, emotions, and skills used over the previous week (Linehan, 1999; for example, see p. 185). The diary card is used to elicit content that will provide therapists with a sense of how target behaviors manifest in a client’s life, as well as to identify patterns of behavior (Linehan, 1999).

Depending on the number and frequency of integration sessions that follow the dosing session phase, an adapted diary card may be of clinical utility to clinicians. If a client identifies new behaviors they want to develop or goals they want to achieve, these could be usefully monitored on a diary card and systematically targeted. Furthermore, ongoing problems that have not resolved during dosing sessions could be monitored and subjected to chain analyses (see below). Whether or not diary cards specifically are employed, the CBT principle of checking in on the previous session’s action plans at the start of a session is key to communicating that action plans are important and to determining the focus of the current session.

#### Chain Analysis

Whereas the diary card provides an overview of behavior, chain analysis is a DBT strategy which allow clinicians to focus in on discrete events (Linehan, 1993). It involves visually depicting the sequence of events (both internal and external) that led up to a target behavior, as well as its consequences (Rizvi and Ritschel, 2014).

Chain Analysis which could be applied to the psychedelic experience itself (although the concept is typically applied to problem behaviors). When it comes to integrating the experiences from the dosing session, it may be worthwhile to use the chain analysis to better understand important or profound moments that participants experience in the weeks and months that follow. Chain analyses may reveal thoughts, behaviors, action urges, and emotions that are associated with these positive changes.

#### Cultivating a Dialectical Stance

At the heart of DBT is a dialectical stance, as a synthesis of acceptance and change (Rathus and Miller, 2015). This dialectical stance promotes a more expansive and nuanced way to view oneself and the experience of others—-moving from “black or white” thinking to “both-and” thinking (Rathus and Miller, 2015, p. 160).

There are numerous apparent paradoxes that can be involved in psychedelic experience, which may be targets of integration sessions. These might include non-ordinary *and* ordinary experience, the profound *and* the mundane, those who “get it” *and* those who don’t, urges to quit jobs or leave relationships that are unfulfilling *and* the need to support oneself and connect with others. A dialectical stance is a useful orientation toward challenges such as these as it allows participants to explore goal states while accepting and validating where they currently are in their lives.

### Acceptance and Commitment Therapy

#### Metaphor

An emphasis on experiential forms of learning in ACT leads to a clinical tool that is frequently used: experiential exercises and metaphor (Bennett and Oliver, 2019). Villatte et al. (2014) propose that “the story-like quality of metaphors has the advantage of providing instructive lessons that are rich in emotional and perceptual detail, mimicking direct contact with the environment and making the experience more memorable” (p. 17).

Clinicians might benefit from incorporating some of the metaphors that have come out of ACT into integration sessions. Psychedelic experience can be difficult to put into words, or *ineffable* (e.g., Yaden et al., 2016). Thus, the use of metaphor and experiential exercises is a way of helping to integrate an experience that is beyond words using therapeutic approaches that are also meant to go beyond words. For example, spontaneously visual images that merge during psychedelic sessions could be utilized in ACT as a guide for future behavior without necessarily having to fully understand what the image “means.”

#### Self-as-Context

Self-as-context refers to “a continuous and secure ‘I’ from which events are experienced, a self that contains but is also distinct from those events” (Luoma et al., 2017, p. 28). Other terms for self-as-context are self-as-perspective, flexible perspective taking, the observing self, pure awareness, or the transcendent self (Luoma et al., 2017). This more flexible and responsive sense of self contrasts with the *conceptualized self*, which includes all the historically derived and verbally constructed self-concepts that are inherently restricting (Hayes et al., 2012).

Clinicians might call upon this concept in integration sessions. Contact with an observing sense of self that is already inherently integrated can provide a stable place from which to observe and process the alterations in sense of self and other that can occur during psychedelic sessions. This allows participants flexibility in regard to which self-concepts (or self-stories) work for them and which interfere with their value driven life. Theory related to self as context can also guide therapists on how to work with alterations of the sense of self, such as reports of “ego dissolution” (Nour et al., 2016; Yaden et al., 2017a) that occur during psychedelic sessions. Furthermore, this process provides a way to work with reports of encounters with external entities or divinities (e.g., Yaden et al., 2017b; Griffiths et al., 2019; Davis et al., 2020b) or perceptions related to the nature of consciousness (e.g., Yaden et al., 2021c) that does not entail taking a stance on whether such experiences are “real” or not (for an extended discussion, see Yaden and Newberg, in press).

#### Committed Action

Committed Action is the key change process in ACT and is defined as “values-based action” (Hayes et al., 2012, p. 328). Hayes (2019, p. 328) put it this way, “if a client does not change his or her behavior, then all of our efforts working on defusion-acceptance, present moment-self-as-perspective, and values are for naught.”

Committed action in psychedelic therapy could look like sticking with a challenging experience in session, allowing oneself to be vulnerable, returning for all of the integration sessions, or making changes in one’s life that make it more fulfilling and aligned with one’s values. For example, if a patient with alcohol use disorder seeks to cut back on their drinking in order to be more present with their family, they might take make a schedule of just how much and when they will cut back on their drinking over the coming week and then follow that schedule, in service of their longer-term goal and their value of family. The whole point of cultivating psychological flexibility, ultimately, is to be able to use it as a tool to live more fully. This concept (and change process) is of great value in psychedelic therapy, where the sometimes-profound experiences had during psychedelic sessions may not automatically result in lasting behavior change.

## Discussion

We have provided a review of historical, sociological influences on contemporary psychedelic psychotherapy as it is practiced largely in clinical healthcare research settings and have argued that cognitive-behavioral frameworks (i.e., CBT, DBT, and ACT) should be considered the default. That said, to the degree that some investigators choose to use other approaches, we should evaluate outcomes, and ultimately, research randomizing individuals to different therapeutic approaches (within ethical limits), as this would provide the most importance evidence on this topic, at least regarding safety and efficacy. We provided rationale largely resting on more empirically founded and testable theory, stronger connection to the evidence base of contemporary science, reduced potential to cause offense, and large amount of safety and efficacy data across a number of treatment contexts.

There are other frameworks that we have not discussed in great detail here but deserve mention and some discussion, these include motivational interviewing, emotion-focused therapy, and supportive psychotherapy. Motivational interviewing (MI) emerged from the research on addiction and is defined as “a collaborative conversation style for strengthening a person’s own motivation and commitment to change” (Miller and Rollnick, 2012, p. 12). Rather than targeting change processes, MI seeks to prepare clients for change by guiding a conversation that ultimately encourages clients to be engaged, empowered, open, and understood (Miller and Rollnick, 2012). MI has been used in at least one clinical trial with psilocybin (Bogenschutz et al., 2015). We believe motivational interviewing could be used as an adjunct intervention. However, we do not believe motivational interviewing is broad enough to be a comprehensive treatment approach for many disorders or difficulties that present as part of psychedelic assisted therapy.

Emotion-focused therapy is a therapy approach emerging from the humanistic tradition that views emotions as centrally important in the experience of the self, in maintaining both adaptive and maladaptive functioning, and in the therapeutic change process (Greenberg, 2011). It has been empirically studied for depression, social anxiety, complex trauma, generalized anxiety, and eating disorders (Goldman, 2019), but the evidence base for this approach is not nearly as extensive as for CBT, including specifically in the context of psychedelics.

The default paradigm currently used in clinical trials with psychedelics is overtly something like supportive psychotherapy, as it is generally characterized as empathetic in a non-directive manner (e.g., Winston et al., 2004). Arguably, this should not change. However, we believe that supportive psychotherapy consists of a set of clinical practices into which concepts from other frameworks invariably slip in. In other words, we believe that many of the clinicians, guides, and monitors who are overtly providing supportive psychotherapy in psychedelic contexts are drawing from an eclectic blend of the other influences on psychedelic psychotherapy that we have already reviewed. To the extent that this is the case, we argue that drawing more explicitly from concepts from cognitive-behavioral approaches (e.g., CBT/DBT/ACT) is advisable.

## Conclusion

We have argued that CBT approaches have the strongest rationale to be the default option for a psychotherapeutic paradigm to pair with psychedelic treatments in mainstream American and European clinical research contexts. We examined some common alternatives and found that they each have problems that are absent or substantially reduced in CBT approaches. We have also provided a substantial number of concepts from CBT, DBT, and ACT that appear relevant to psychedelic treatments. While we believe cognitive-behavioral approaches should be the default in psychedelic psychotherapy, we are open to and supportive of additional scholarship and research on the other approaches considered here as well as others. Furthermore, the CBT/DBT/ACT concepts listed are provided for illustrative purposes and are not meant to be comprehensive and should be subjected to further research. Overall, we believe participant and patient safety and efficacy should be paramount considerations in psychedelic treatments and we believe cognitive-behavioral approaches currently best fulfill these criteria.

## Author Contributions

DY conceived the project and wrote the manuscript. DE and MG conducted literature reviews and provided writing. DF-W provided writing and edits. JL and MJ provided writing and edits. All authors contributed to the article and approved the submitted version.

## Conflict of Interest

MJ was an advisor to the following organizations regarding the medical development of psychedelics and related compounds: AJNA Labs LLC, AWAKN Life Sciences Inc., Beckley Psychedelic Ltd., Entheon Biomedical Corp., Field Trip Psychedelics Inc., Mind Medicine Inc., and Otsuka Pharmaceutical Development & Commercialization Inc. The remaining authors declare that the research was conducted in the absence of any commercial or financial relationships that could be construed as a potential conflict of interest.

## Publisher’s Note

All claims expressed in this article are solely those of the authors and do not necessarily represent those of their affiliated organizations, or those of the publisher, the editors and the reviewers. Any product that may be evaluated in this article, or claim that may be made by its manufacturer, is not guaranteed or endorsed by the publisher.

## Footnotes

1 Nayak, S. M., Singh, M. Yaden, D. B., and Griffiths, R. R. (in preparation). *Belief Changes Associated With Psychedelic Use.*
